The article "Analysis of the Rare Earth Mineral Resources Reserve System and Model Construction Based on Regional Development" was published in 2022. Journal: Comput Intell Neurosci.

# Analysis of the Rare Earth Mineral Resources Reserve System and Model Construction Based on Regional Development

**DOI:** 10.1155/2022/9900219

**Published:** 2022-07-04

**Authors:** Dafang Shi, Shouting Zhang

**Affiliations:** China University of Geosciences (Beijing), Beijing 100191, China

## Abstract

China is a large rare earth country that has pushed for related rare earth research, development, and application in the global development and progress of rare earths. The rare earth resource reserve strategy must be implemented by China due to the situation of rare earth resources at home and abroad, national security, and the need to strengthen the right to speak in the international market. This article builds the rare earth mineral resources reserve system and model from the perspective of regional development and uses the improved SURF algorithm to solve the problems of inaccurate mine location, mine location deviation, dislocation, overlap, and other issues, resulting in more accurate mineral resources reserve management data. The results show that the maximum relative error between the parallel profile method and the traditional method is 2.6%, which meets the requirement for mineral reserve calculation accuracy and can be used to calculate reserves. China's peak ionic rare earth output will be 46,797.06 tonnes in 2024, and then, it will decline at a 4% annual rate thereafter. This demonstrates how a graded reserve and orderly promotion can improve the workflow and efficiency of the rare earth mineral resources reserve.

## 1. Introduction

China has the world's richest proven rare earth reserves, and the variety, quality, output, and export of rare earths frequently rank first in the world [1, 2], making it critical to the global rare earth supply. China is a large rare earth country that has pushed for related rare earth research, development, and use in the global development and progress of rare earths. However, environmental damage, backward technology, low technological content of products, excessive export, low price, indiscriminate mining and excavation, and other serious issues plague China's development and utilization of rare earth resources.

Modeling of reserves: A steady supply of resources is critical whether it is for national economic security or national defence security. To begin with, a country's economic development is heavily reliant on resources, particularly strategic resources, and the economy's long-term viability cannot be separated from a reliable supply of resources. In modern industry [3], high-tech, and national defence technology, rare earth is an essential strategic mineral resource. Pan et al. believed that there have been many studies on the catalytic and surface performance of alkali metal, alkaline earth metal, and other metal oxides, but rare earth oxides have received relatively little attention [4]. Krishnamurthy presented and explained the geochemical characteristics, classification, and distribution of rare earth elements in sedimentary rocks [5]. Xiao investigated the effect of rare earth elements on the compressive ductility of ferromagnetic shape memory alloys and found that rare Earth elements can significantly improve the material's compressive ductility [6]. According to Ilyas et al., the output of foreign rare earths will increase significantly due to the restart of rare earth projects in countries other than China and the expansion of related rare earth enterprises [7]. Rare earth is a crucial component of modern weapons and equipment. To ensure national sovereignty and protect against foreign invasion, rare earth must be preserved. As a result, we can only ensure domestic demand for a sustainable supply of rare earth and national defence security by reserving rare earth and other strategic resources and increasing the degree of protection of rare earth resources.

The article "Analysis of the Rare Earth Mineral Resources Reserve System and Model Construction Based on Regional Development" was published in 2022. Journal: Comput Intell Neurosci.

The research on the optimal allocation of rare earth resources is conducive to solving the problems existing in the development and utilization of rare earth resources, improving the economic and social benefits of rare earth resources development, contributing to the healthy and sustainable development of rare earth industry, and having important practical significance for the optimization of regional development economic layout structure and the implementation of national rare earth strategy [8]. At the same time, the research on this topic also has reference significance for the research of other important mineral resources optimal allocation.

The main innovations of this article are as follows:

1. The reserve system of rare earth mineral resources oriented to regional development has been constructed, and the quantitative evaluation standards of some indexes have been established, which not only helps to improve the scientificity and accuracy of index evaluation but also provides a reference for the research of other resources' optimal allocation.
2. Aiming at the characteristics of a large matching area and high precision of mine spatial location, the SURF algorithm is improved in the order of feature point extraction, pixel optimization in the feature extraction stage, and image segmentation in the feature extraction process.
3. The clustering results of geochemical sampling points by K-means have a corresponding relationship with the stratigraphic lithology distribution in the corresponding sampling areas, and clustering can achieve good geological results. Graded reserve and sequential advance can clarify the workflow and improve the work efficiency of rare earth mineral resources reserve.

The article "Analysis of the Rare Earth Mineral Resources Reserve System and Model Construction Based on Regional Development" was published in 2022. Journal: Comput Intell Neurosci.

The section structure of this study is as follows: Section 1 introduces the research background and significance and then introduces the main work of this article.  Section 2 mainly introduces the related research status of rare earth mineral resources.  Section 3 puts forward the specific methods and implementation of this research.  Section 4 verifies the superiority and feasibility of this research model.  Section 5 is the summary and prospect of the full text.

## 2. Related Work

### 2.1. Research on Rare Earth Resources

Rare earth is of great strategic value. With its abundant rare earth resources and cheap production cost, China has achieved the first output, the first application, and the first export in the world rare earth resources. Nassani et al. pointed out that the current supply cost of rare earths is too low, and the supply of rare earths far exceeds the demand, which is an important reason for the low price of rare earths [9]. Li and Peng pointed out that there are some problems in China's rare earth industry, such as waste of resources, environmental pollution, unreasonable product structure, lagging development of end products, and imperfect quota management. They put forward some measures to promote the development of China's rare earth industry, such as strengthening the source control of rare earth, strengthening the research of rare earth application theory, and perfecting quota management [10].

Raharjo et al. think that the government should strengthen the management and protection of rare earth resources, actively guide enterprises to develop into high-end application industries, and increase the economic added value of industries, so as to promote the sustainable development of rare earth industry and improve its competitiveness in the international market [11]. Gromov et al. focused on the storage and exploitation status of rare earth resources. On the basis of the research on the whole rare earth resources, they found that there were some problems in the rare earth industry, such as serious resource waste, severe environmental pollution, and chaotic industry supervision, and put forward some measures to improve the utilization efficiency of rare earth resources and turn the advantages of rare earth resources into economic advantages [12]. Diether et al. thought that the upstream and downstream enterprises of rare earth industry are all self-interested, and the main bodies in the industry chain are in their own way, and there is no sufficient information communication between them, ignoring the government's policy guidance, which leads to the low comprehensive performance of the rare earth industry chain [13]. Zhai et al. studied the important role of rare earth in iron and steel production and pointed out that rare earth elements can improve the shape and distribution of inclusions, refine grains, and then significantly improve the impact toughness, tensile strength, and oxidation resistance of products [14].

The article "Analysis of the Rare Earth Mineral Resources Reserve System and Model Construction Based on Regional Development" was published in 2022. Journal: Comput Intell Neurosci.

### 2.2. Research on Optimal Allocation of Resources

Optimal allocation of resources is the core topic of economic research, which can be summarized as static allocation and dynamic allocation of resources in terms of methodology. Norregaard et al. studied the optimal utilization of exhaustible resources by a mathematical model and pointed out that if the social value of nonrenewable resources is to be maximized, the price growth rate of the resources should be equal to the discount rate [15]. Chen et al. have made a long-term and in-depth study on the optimal depletion path and capital accumulation of nonrenewable resources [16]. Fu et al. thought that the mining industry is facing many severe sustainability challenges and studied and constructed the indicator system framework of sustainable development of the mining industry, which includes economic, environmental, social, and comprehensive indicators [17]. Liu et al. deeply studied the physical and chemical properties of rare earth elements and discussed the related applications of rare earth elements in catalytic materials, permanent magnet materials, hydrogen storage materials, luminescent materials, and agriculture [18].

Wang et al. systematically summarized the utilization status and broad prospects of rare earth elements in tricolor fluorescent lamps, electroluminescent materials, and fluorescent materials for medical devices. At the same time, they also pointed out that there was still a big gap between the application level of rare earth elements in China and some foreign countries [19]. Shibuya et al. elaborated the process and polishing mechanism of polishing powder, focused on the application fields of polishing powder, and looked forward to the future application of products [20]. Liu et al. thought that the total amount of nonrenewable mineral resources in the crust is a fixed value, but the economically recoverable reserves change dynamically with time. Liu et al. discussed how to use the market mechanism to optimize the allocation of mineral resources under the market economy [21].

## 3. Research Method

### 3.1. Rare Earth Mineral Resources Reserve System

The crust is rich in rare earth elements, but they are scattered. As a result, although rare earth elements have vast absolute reserves, there are currently few rare earth minerals that can be used in industrial production, and they are also unevenly distributed around the globe. Whether it is Japan, the European Union, or other major rare earth consumer countries, or the United States, Russia, India, Australia, and other major rare earth producers and consumers, they have recognized the strategic position and importance of rare earth mines, formulated relevant laws and regulations, established a rare earth resource strategy that is appropriate for their own economic development, and made arrangements and arrangements for the production and consumption of rare earths. Many countries' practises in this area have significant reference significance for China's rare earth development and are worthy of in-depth study and enlightenment by relevant Chinese departments and experts in order to improve China's rare earth resource strategy.

The article "Analysis of the Rare Earth Mineral Resources Reserve System and Model Construction Based on Regional Development" was published in 2022. Journal: Comput Intell Neurosci.

Because a large portion of the areas where rare earth resources are reserved are rare earth mining provinces, these areas with rare earth industry as the pillar and local rare earth resources as the main source of fiscal revenue, once the reserve of rare earth resources is implemented, it will reduce the income from resource development in rare earth resources reserve areas, causing local economic backwardness. As a result, it is important to understand how central interests and local interests can be reconciled, taking into account the stark contradiction between rare earth resources and mineral reserves and local development, and ensuring that local economic interests are not jeopardized and social development is stable, which is also a major impediment to China's implementation of strategic rare earth resource reserves.

The research results of optimal allocation and protection zoning of rare earth resources serve the practice of mineral resources planning, which determines the practicability of the research method. It is the working principle of this study to adopt the principle research method that the optimal allocation of empirical rare earth resources should strictly implement the access conditions of technology and environmental protection. China is rich in rare earth resources, and there are great differences in rare earth ore reserves, types, grades, and industrial basic conditions for regional development in different regions. These differences determine the differences in the initial conditions for developing rare earth resources and developing economy in different regions. The analysis and research of these differences can make a scientific evaluation of the resource elements for developing different regions.

The article "Analysis of the Rare Earth Mineral Resources Reserve System and Model Construction Based on Regional Development" was published in 2022. Journal: Comput Intell Neurosci.

The development and utilization of rare earth resources, as well as their optimal allocation and other activities, must be carried out not only in accordance with the characteristics of the resources, the level of regional industrial development, and other factors but also in accordance with a number of constraints. The resource development and utilization constraint index is a negative factor. The greater the impact on resource development, utilization, and allocation, the stronger the constraint. The smooth development of rare earth resources is directly linked to the degree of water security and water cost. The cost of land use in the early stages of resource development, which primarily affects mining areas that have not yet begun construction or large-scale expansion, is known as land resource constraint. The cost of developing rare earth resources or destroying other resources is known as other resource constraints. The cost constraint becomes more severe as the cost rises. The index hierarchy of the evaluation index system is shown in Figure 1.

The geographic location, geometric shape, and reserve information of mineral resources are the key points of mineral resources management [4]. Three-dimensional geological models established by mining software are mainly divided into three categories: exploration engineering database, geological entity model, and reserve block model. Then, based on the standards, the coordination of modeling and design of geological survey and mining is realized, and a unified process and standardized model data are formed. Through the execution management of geological survey production, the sequential and real-time geological survey data can be realized so as to realize the three-dimensional dynamic management of mineral resources reserves. The construction framework is shown in Figure 2.

The digital standard provides the foundation for managing rare earth mineral resources digitally. Mine geological survey digital standards include technological standards, production and operation standards, data standards, and geological survey knowledge base, which involve geological modeling and model updating, reserves estimation and statistics, and actual measurement modeling and statistics. The fine management of the entire process of mineral resources by mines and mining groups can be realized, and the dynamic integrated management of geological exploration reserves, production reserve, mineral production consumption, and resource reserve can be realized by systematically guiding the planning management of mine geological exploration and mining production.

The article "Analysis of the Rare Earth Mineral Resources Reserve System and Model Construction Based on Regional Development" was published in 2022. Journal: Comput Intell Neurosci.

The digitized and informationized technological process of geology, survey, and mining underpins the collaborative platform for geological survey and mining. It can streamline and standardize 3D digital modeling and design by allowing real-time data sharing and collaborative operation on the same platform and environment. Change the traditional technical mode, lowering labour intensity and production costs while increasing technician productivity and quality.

### 3.2. Classification of Reserve Levels

There are basically two forms of mineral resources reserves in the world: mineral products reserves and mineral resources strategic base reserves. Comparatively speaking, the reserve cost of mineral resources strategic base is low, and the reserve is safe. The disadvantage is that it takes a long period to use, and it has a weak ability to reflect short-term supply interruption and price changes. The reserve cost of mineral products is high and the operation and management are complicated, but its advantage is that it can be put into the market quickly to ensure timely supply.

Mineral resources are strategic base reserves, the object of reserves is the areas that contain or may contain important strategic minerals, and in fact, the reserves are proved reserves or unexplored resources. The operation of other metal mineral resources reserves and the management of mineral resources can also refer to the practice of oil to establish product reserves. It should be noted that it is necessary to select the reserve of mineral resources strategic base, raw material type or product type reserve, or both in combination with specific minerals.

A strategic reserve is the reserve of mineral land to prevent the shortage of resources caused by unexpected events or uncertain factors and ensure the sustainable supply of the mineral resources in China. In order to improve the reliability of *T* value, the average value of historical survey data of several discovered resource sites is used to express it.

(1) $$\begin{array}{c} T=t_{\text{generalsurvey}}+t_{\text{siftthrough}}+t_{\text{explore}}. \end{array}$$

Then the reserve scale model of strategic reserve can be established as shown in the following formula:

(2) $$\begin{array}{c} R_{1}=\sum_{i=1}^{n}\frac{C_{i}^{1}}{\alpha }, \end{array}$$

where *R*_1_ is the scale of strategic reserve; *C*_*i*_^1^ is the domestic consumption in *i* year after the reserve starts; *α* is the comprehensive utilization rate of resources, which is the product of mining recovery rate and mineral processing recovery rate.

Advantage reserve is to prevent the worldwide resource shortage caused by unexpected events or uncertain factors and to ensure the sustainability of the advantage of mineral resources in advantage strategy. It must be emphasized that the reserve can meet the consumption of this mineral in foreign *T* time, which is not the same as having to meet foreign demand but only as a strategic bargaining chip of the country when resources are in short supply. Therefore, the scale model of the advantageous reserve can be established, as shown in the following formula:

(3) $$\begin{array}{c} R_{2}=\sum_{i=1}^{n}\frac{C_{i}^{2}}{\alpha }, \end{array}$$

where *R*_2_ is the advantageous reserve scale; *C*_*i*_^2^ is the consumption of this mineral product in the world except China in *i* year after the reserve starts; *α* is the comprehensive utilization rate of resources.

The article "Analysis of the Rare Earth Mineral Resources Reserve System and Model Construction Based on Regional Development" was published in 2022. Journal: Comput Intell Neurosci.

When calculating the volume of ore bodies in blocks, a reasonable calculation formula should be selected according to the geometric shape and relative area ratio of ore bodies in two adjacent sections, and there are usually the following situations.

When the shapes of two adjacent sections are similar and the relative area difference between them is less than 40%, the block volume is calculated by the trapezoidal formula:

(4) $$\begin{array}{c} V=\frac{1}{2}l\left(S_{1}+S_{2}\right). \end{array}$$

When the shapes of two adjacent sections are similar, but the relative difference of their areas is greater than or equal to 40%, the section cone formula is used to calculate the block volume:

(5) $$\begin{array}{c} V=\frac{1}{3}l\left(S_{1}+S_{2}+\sqrt{S_{1}S_{2}}\right). \end{array}$$

In the above formulas, *V* is the ore body volume of the block, m^3^; *l* is the distance between two sections, *m*; *S*_1_*S*_2_ is the area of the ore body on the block in two adjacent sections, m^2^.

The ore reserves of ore blocks are equal to the volume of ore blocks multiplied by the average weight of ore, which is calculated by the following formula:

(6) $$\begin{array}{c} Q=VD, \end{array}$$

where *Q* is the ore reserve of ore block, *t*; *V* is the ore body volume of ore block, m^3^; *D* is the average ore weight of the ore block, and t/m^3^. *D* is replaced with the arithmetic average of the weights of two sections.

### 3.3. Establishment of the Mathematical Model of Reserve Scale

Rare earth resource reserves cannot be sustained without significant reserve fund investment. The reserve fund is a hybrid of a national reserve fund and a private reserve fund, comprising both the government-backed reserve fund and a large number of privately raised funds. Despite the fact that the gap between China's economic development and that of developed countries around the world is gradually closing, the conditions for rare earth resource reserves are currently met. The author believes that adopting independent legislation for rare earth resource reserves is more appropriate and that China's reserve legislation system will continue to improve as the reserve system is implemented and the economy develops.

The article "Analysis of the Rare Earth Mineral Resources Reserve System and Model Construction Based on Regional Development" was published in 2022. Journal: Comput Intell Neurosci.

SURF (Speeded-Up Robust Features) is a “high robustness” and “high stability” local image feature point detection and matching algorithm, which has few requirements and conditions for image matching. SURF algorithm has been widely used in military reconnaissance, traffic management, face recognition, target detection and tracking, image matching, and many other fields [10].

Assuming a point *p*(*i*, *j*) of an image *f*(*x*, *y*), on the scale *σ*, the Hessian matrix *H*(*x*, *σ*) of this image is defined as follows:

(7) $$\begin{array}{c} H\left(x,\sigma \right)=\left[\begin{array}{cc} L_{XX}\left(X,\sigma \right) & L_{XY}\left(X,\sigma \right)\\ L_{XY}\left(X,\sigma \right) & L_{YY}\left(X,\sigma \right) \end{array}\right]. \end{array}$$

Among them, *L*_*XX*_ is the convolution of the second derivative of the Gaussian template and image *f*(*x*, *y*) at point *p*(*i*, *j*). When the local value of the Hessian determinant is the largest, we think that the value we seek is the feature point of the image, and its *L*_*XX*_, *L*_*YY*_ is the same.

When SURF calculates the feature point information of the image, a 3D template is used. According to the preset Hessian matrix threshold *H*, when *h* > *H*, the points that are larger than the response values of 26 adjacent points are selected as the interest points [12]. Finally, the position of the feature points is accurately determined by interpolation.  Figure 3 shows the interpolation diagram.

However, the traditional SURF algorithm still has its shortcomings, especially when the algorithm calculates the main direction of feature vectors, it has certain limitations. For example, some images have higher exposure, while others have lower exposure. Therefore, in view of the characteristics and shortcomings of the traditional SURF algorithm in the geoscience field, this article optimizes and improves the matching of mine DEM (digital elevation model).

In this matching work, the edge of the image is protected by using the advantages of the bilateral filter. At the same time, the filter filters out a large amount of image noise, which avoids the result of matching failure caused by multisource and multitemporal imaging methods. The following is the mathematical expression of the bilateral filtering method:

(8) $$\begin{array}{c} H_{BL}\left(I_{x}\right)=\frac{1}{W_{X}}\sum_{y\in s}G\sigma_{d}\left(\left\|x-y\right\|\right)G\sigma_{\gamma }\left(I_{x}-I_{y}\right)I_{y}. \end{array}$$

Among them,

(9) $$\begin{array}{c} W_{X}=\sum_{y\in s}G\sigma_{d}\left(\left\|x-y\right\|\right)G\sigma_{\gamma }\left(I_{x}-I_{y}\right). \end{array}$$

*K*-means is a commonly used partition-based clustering method [22], which is used to group samples according to the similarity between sample attribute values. *K*-means is regarded as an unsupervised classification method. The basic idea is to divide the data set into *K* classes, and the samples in each class are very similar, but the samples in different classes are very different.

The article "Analysis of the Rare Earth Mineral Resources Reserve System and Model Construction Based on Regional Development" was published in 2022. Journal: Comput Intell Neurosci.

In each iteration of the algorithm, each sample is assigned to the class represented by the nearest centroid. The distance is expressed by the square of Euclidean distance, so the distance from sample *i* to centroid *j* is as follows:

(10) $$\begin{array}{c} d_{ij}={\left\|X_{i}-C_{j}\right\|}^{2}={\sum_{q=1}^{Q}\left(X_{qi}-C_{qi}\right)}^{2}, \end{array}$$

where *X*_*i*_ is the vector composed of attribute values of sample *i*, *C*_*j*_ is the centroid vector of class *j*, *Q* is the number of attributes, *X*_*qi*_ is the *q* attribute value of the *i* th sample, and *C*_*qi*_ is the *q* attribute value of the centroid of class *j*.

For each sample, calculate its distance from each centroid. The record is assigned to the class whose centroid is closest to the record. In this process, a sample may be transferred from one class to another.

Taking geochemical sampling points as data objects, geochemical elements of sampling points as attributes, and element analysis results as attribute values, K-means is used for clustering analysis. Get the category characteristics of each sample and the average value and standard deviation of each category. The purpose of cluster analysis is to study the distribution characteristics and laws of regional geochemical elements and find meaningful resource targets.

When *K*=7, the correlation analysis is carried out on the data of one area, and the correlation coefficients among 25 groups of element samples are obtained. After *r* < 0.3, the elements are connected with each other, and no research is done. Generate the correlation analysis linear graph, as shown in Figure 4.

There is a certain gap in the correlation results due to the difference in the five correlation data of *k* as 7,8,9,10, and 11. We take the correlation analysis results that have the same majority; that is, La is related to Pr, Nd is related to Pm, Eu is related to Gd, Tb, and Er is related to *Y*.

## 4. Result Analysis

Taking a rare earth mine as an example, this article introduces how to use the parallel section method to estimate resource reserves in DIMINE software. DIMINE software can calculate the mine reserves and then calculate the mine metal quantity according to the average grade of each block. In this article, the calculation data of four blocks are selected and calculated by the traditional reserve estimation method and the parallel section method, respectively. The calculation results are given in Table 1. The calculation results of the two methods are analyzed and compared, and the comparison results are given in Table 2.

The article "Analysis of the Rare Earth Mineral Resources Reserve System and Model Construction Based on Regional Development" was published in 2022. Journal: Comput Intell Neurosci.

The results of the calculations show that the maximum relative error between the parallel section method and the traditional method is 2.6 percent, which meets the requirements for mineral reserve calculation accuracy and can be used to calculate reserves. This demonstrates that the parallel section method can be used to estimate mine reserves. This method improves not only the working efficiency of reserves estimation but also the visual analysis degree of reserves estimation to some extent.

Based on the output data of ionic rare earths, we choose the annual data with a good linear relationship and use the linear trial and error method to calculate and predict the future output of mixed rare earths. The forecast results show that the peak output of ionic rare earths in China will appear in 2024, with a peak output of 46,797.06 tons, and then it will decrease at an average annual rate of 4% (Figure 5).

Rare earth is the general name of a group of elements, including La, Ce, Pr, and Nd, which mostly occur in the form of rare earth oxides. Due to the differences in the electronic layer structure and physical and chemical properties of each element atom, the application fields of different elements are also different. From the forecast results, the oxides of each element show different growth trends and peak output (Figure 6).

Mixed rare earth and bastnaesite output has reached or will soon reach a peak, owing to the fact that the minerals containing light rare earth are primarily mixed rare earth and bastnaesite, whereas ionic rare earth output is steadily increasing. It is because only ion adsorption minerals and xenotime contain heavy rare earths, and they are mostly concentrated in southern China. As a result, the world's heavy rare earths (such as terbium, erbium, dysprosium, and yttrium) are primarily supplied by ion adsorption rare earth mines in southern China, and this pattern cannot be significantly improved in a short period of time, and China retains its monopoly advantage.

In order to verify the practicability of the SURF algorithm in mine spatial location determination, this article designed a verification test to verify the robustness of the algorithm. We used several rare earth mines as experimental objects and carried out matching experiments from different angles. The verification results of the mine positioning effect are shown in Figure 7.

The article "Analysis of the Rare Earth Mineral Resources Reserve System and Model Construction Based on Regional Development" was published in 2022. Journal: Comput Intell Neurosci.

As can be seen from Figure 7, only one of the seven different types of mines selected from the database under different geological conditions failed to identify their spatial positions, and the other six mines could identify the feature points to be matched with high accuracy. We began to study when *k* took 3, and the research value below 3 was not significant. The value of *K* determines how many sampling points (data objects) we classify. The purpose of choosing different *K* values is to analyze the stability and reliability of clustering results. The quality report generated by *K*=4 ~ 10 is shown in Figures 8–10.

The red background area in the class similarity report indicates that the similarities between classes are very close, the yellow background area indicates that the similarities between classes are not far or near, and the green background area indicates that the similarities between classes are far. The clustering segmentation is considered strict when most or all of the background colours are green, and the clustering effect is excellent because there is sufficient separation between classes. The absence of a red background indicates that the clustering result is satisfactory. When *K* is greater than 10, although the intraclass deviation is small, the interclass deviation is large. However, the red and yellow background increased, while the green background decreased. It shows that the clustering effect begins to decline. Therefore, in this topic, we only study the K-means clustering analysis with *K* from 4 to 9. The clustering effect is better according to the summary of the quality report generated by clustering. It conforms to the basic idea of clustering: make the similarity of samples within the class as large as possible and the similarity of samples between classes as small as possible.

## 5. Conclusion

Due to their unique physical and chemical properties, rare earths are widely used in national economic development, national defence, and military construction. This article analyzes the current situation and existing problems of rare earth resources development and utilization in China and constructs a rare earth mineral resources reserve system based on research on the construction of rare earth mineral resources reserve system and model based on regional development. The reserves of rare earth mineral resources are divided into different levels of mineral reserves, including strategic reserves, dominant reserves, and controlled reserves, according to different levels of strategic objectives, and corresponding mathematical models of reserves scale are established for strategic reserves and dominant reserves. The maximum relative error between the parallel profile method and the traditional method is 2.6 percent, which meets the precision requirement of mineral reserve calculations and can be used to calculate reserves. China's peak ionic rare earth output will be 46,797.06 tonnes in 2024, and then, it will decline at a 4% annual rate thereafter. The stratigraphic lithology distribution in the corresponding sampling areas has a corresponding relationship with the K-means clustering results of geochemical sampling points. Clustering has the potential to improve geological effect and geochemical exploration efficiency.

The article "Analysis of the Rare Earth Mineral Resources Reserve System and Model Construction Based on Regional Development" was published in 2022. Journal: Comput Intell Neurosci.

## Figures and Tables

**Figure 1:** Index hierarchy chart of the evaluation index system.

**Figure 2:** Construction framework of dynamic management of rare earth reserves.

**Figure 3:** Construct scale space map.

**Figure 4:** Data correlation analysis linear graph.

**Figure 5:** Prediction of rare earth ore yield.

**Figure 6:** Output prediction of each element oxide.

**Figure 7:** Verification result of the mine positioning effect.

**Figure 8:** Class deviation comparison.

**Figure 9:** Class distribution comparison.

**Figure 10:** Class similarity comparison.

**Table 1:** Block reserves calculation.

Method	Block name	Segment volume (m^3^)	Volumetric weight of ore (tm^−3^)	Mineral resources (t)	Block grade (%)	Rare earth quantity (t)
Traditional method	A1-21	8736.21	2.88	2213.71	0.55	141.21
	A2-22	5886.01	2.88	1628.93	0.63	102.37
	A3-23	996.27	2.88	2849.72	0.87	22.17
	A4-24	7896.62	2.88	2214.66	0.66	140.61
Parallel section method	A1-21	8512.71	2.88	2336.89	0.56	142.47
	A2-22	6003.87	2.88	19632.25	0.81	147.25
	A3-23	1022.41	2.88	2886.91	0.89	116.85
	A4-24	8201.93	2.88	20124.76	0.64	66.89

**Table 2:** Comparative analysis of block reserves calculation.

Block	Traditional method	Parallel section method	Contrast (%)
A1-21	8736.21	8512.71	2.6
A2-22	5886.01	6003.87	2
A3-23	996.27	1022.41	2.6
A4-24	7896.62	8201.93	3.9

## Data Availability

The data used to support the findings of this study are available from the corresponding author upon request.
